The article "On Improved 3D-CNN-Based Binary and Multiclass Classification of Alzheimer's Disease Using Neuroimaging Modalities and Data Augmentation Methods" was retracted in 2023. Reasons: signs of a paper mill; suspected computer-generated content; unreliable results or conclusions; concerns about the data.

# On Improved 3D-CNN-Based Binary and Multiclass Classification of Alzheimer's Disease Using Neuroimaging Modalities and Data Augmentation Methods

**DOI:** 10.1155/2022/1302170

**Published:** 2022-02-11

**Authors:** Ahsan Bin Tufail, Kalim Ullah, Rehan Ali Khan, Mustafa Shakir, Muhammad Abbas Khan, Inam Ullah, Yong-Kui Ma, Md. Sadek Ali

**Affiliations:** ^1^School of Electronics and Information Engineering, Harbin Institute of Technology, Harbin 150001, China; ^2^Department of Electrical and Computer Engineering, COMSATS University Islamabad Sahiwal Campus, Sahiwal, Pakistan; ^3^Department of Zoology, Kohat University of Science and Technology, Kohat 26000, Pakistan; ^4^Department of Electrical Engineering, University of Science and Technology Bannu, Bannu 28100, Pakistan; ^5^Department of Electrical Engineering, Superior University, Lahore 54000, Pakistan; ^6^Department of Electrical Engineering, Balochistan University of Information Technology,Engineering and Management Sciences, Quetta,Balochistan 87300, Pakistan; ^7^College of Internet of Things (IoT) Engineering, Hohai University (HHU), Changzhou Campus 213022, China; ^8^Communication Research Laboratory, Department of Information and Communication Technology, Islamic University, Kushtia-7003, Bangladesh

## Abstract

Alzheimer's disease (AD) is an irreversible illness of the brain impacting the functional and daily activities of elderly population worldwide. Neuroimaging sensory systems such as Magnetic Resonance Imaging (MRI) and Positron Emission Tomography (PET) measure the pathological changes in the brain associated with this disorder especially in its early stages. Deep learning (DL) architectures such as Convolutional Neural Networks (CNNs) are successfully used in recognition, classification, segmentation, detection, and other domains for data interpretation. Data augmentation schemes work alongside DL techniques and may impact the final task performance positively or negatively. In this work, we have studied and compared the impact of three data augmentation techniques on the final performances of CNN architectures in the 3D domain for the early diagnosis of AD. We have studied both binary and multiclass classification problems using MRI and PET neuroimaging modalities. We have found the performance of random zoomed in/out augmentation to be the best among all the augmentation methods. It is also observed that combining different augmentation methods may result in deteriorating performances on the classification tasks. Furthermore, we have seen that architecture engineering has less impact on the final classification performance in comparison to the data manipulation schemes. We have also observed that deeper architectures may not provide performance advantages in comparison to their shallower counterparts. We have further observed that these augmentation schemes do not alleviate the class imbalance issue.

## 1. Introduction

Alzheimer's disease (AD) is a global health concern associated with pathological changes inside the brain [1–3]. It has an upward trend for increase in people aged 65 or older [4]. Brain regions such as presubiculum, subiculum, fimbria, left pericalcarine, right hippocampus fissure, and inferior lateral ventricular are affected during the progression of AD [5]. Imaging, clinical, biological, and genetic manifestations of AD drive new research [6]. Successful intervention by a medical expert for treatment purposes is dependent on early diagnosis of AD. To capture neurobiological changes occurring during the progression of AD, neuroimaging modalities such as the Magnetic Resonance Imaging (MRI) and Positron Emission Tomography (PET) are routinely applied [7]. Neurofibrillary tangles and amyloid plaque depositions are major hallmarks of AD [8]. Challenges such as high dimensionality limit the performance of discrimination methods of AD.

A number of studies have been reported in the literature for multimodality based discrimination of AD/Mild Cognitive Impairment (MCI) [9], landmark-based feature extraction method to distinguish AD subjects from normal controls (NC) [10], recursively wasting away uninformative features for AD/MCI diagnosis [11], employment of data augmentation techniques for multiclass AD/NC/MCI classification task [12], AD/MCI classification employing data augmentation using stacked autoencoder based features [13], autoencoder based features for NC/MCI classification [14], MCI-to-AD conversion using MRI modality extracting multiple patches for data augmentation in Convolutional Neural Networks (CNN) [15], resting-state eyes-closed electroencephalographic rhythms for AD/NC classification [16], MCI-to-AD alteration by using mechanical MRI data and genetic algorithm [17], combination of deep learning (DL) architectures for MCI/NC and AD/NC classification [18], voxel-based, cortical thickness as well as hippocampus based methods for different classification problems [19], and a manifold-based semisupervised learning approach for NC/MCI classification [20].

In addition, the authors used a 3D convolutional autoencoder for binary and multiclass classification methods [21], deep 3D-CNN for binary and multiclass classification problems [22], utilization of longitudinal structural MR images for AD/NC and MCI/NC classification tasks [23], Gaussian process based MCI-AD conversion prediction [24], amnestic MCI/NC classification using a multivariate method [25], AD/NC classification using deep belief networks [26], an integrated multitask learning framework for different binary classification tasks [27], prognostic model using longitudinal data [28], sparse learning method for different binary classification tasks [29], a grading biomarker using sparse representation techniques for MCI-to-AD conversion [30], framework for different binary classification tasks using hierarchical features [31], inception version 3 transfer learning model for multiclass classification using different data augmentation schemes [32], and using a 3D-CNN architecture for binary classification tasks employing data augmentation methods [33–36].

Data augmentation techniques make DL networks more robust and help them to obtain good performance [37]. Learning invariant features is a nontrivial task [38]. However, many modern CNN architectures are not shift-invariant causing drastic changes in the output which lead to incorrect predictions [39]. The CNN architecture typically ignores the classical sampling theorem [40]. Deep CNN networks show stability against rigid translations [41–44], rotations, or scalings [45, 46] due to their equivariance to small global rotations and translations [47–50]. Rotating the original image by a small factor around its center and then translating it by a few pixels causes the classifier to make a wrong prediction [51–53]. Beside the above studied literature, researchers in academia and industry also investigated other emerging topics in computer and information technology [54–60].

This work aims to study the impact of data augmentation techniques on the early diagnosis of AD. We have used 3D-CNN architectures for feature extraction and classified them into NC, MCI, and AD classes simultaneously as well as bilaterally. We have considered four problems: multiclass classification, among MCI, NC, and AD classes, and binary classifications between MCI and NC classes, MCI and AD, and NC and AD classes. We have studied the impact of three data augmentation methods, such as random width and height shift, random zoomed in/out, and random weak Gaussian blurring, for the early AD diagnosis. We chose these three data augmentation methods over others as their effects are relatively well known and they have been extensively studied in the literature. We worked with limited number of samples to imitate human reasoning model as humans generally require only a few samples of data to learn a task effectively.

Remainder of the paper is organized as follows. In section 2, the datasets considered in this study are described. Methods are described in section 3. Experiments and their results are provided in section 4, whereas section 5 discusses the results. Finally, section 6 draws the conclusions.

## 2. Description of Datasets

In this work, we use MRI and PET scans from the AD Neuroimaging Initiative (ADNI) database. The subject's demographics are given in Tables 1 and 2. The data are split at the subject level for the experimental results.

## 3. Methodology

In this study, we considered four problems: Multiclass (e.g., three classes) classification, among MCI, NC, and AD classes, and three binary classification problems, that is, the binary classification between MCI and NC, MCI and AD, and NC and AD classes. We studied all four problems using the PET dataset, while the MRI dataset is used to study only multiclass and AD/NC binary classification problems. We will now describe the DL architectures for solving these problems using MRI and PET datasets. Furthermore, for the multiclass classification task involving MRI neuroimaging modality, we did not augment samples of MCI class to study the impact of class imbalance on final classification performances.

Detailed multiclass classification architecture employing PET neuroimaging modality and random zoomed (in/out) augmentation is shown in Figure 1. Number of feature maps in convolutional 3D-layer is 6, number of neurons is 100 for Fully Connected (FC) layer 1, 50 for FC layer 2, and 3 for FC layer 3. The input layer takes a volume having size of 79 × 95 × 69.

Figure 1 shows that an input layer is accepting a volume having a size of 79 × 95 × 69. After that, there is a block named block A repeated five times sequentially, with a 3D convolutional layer for feature extraction with a kernel of size 3 in all dimensions, with 6 feature maps and a weight and bias L2 factor of 0.00005 to support in mitigating the impact of overfitting by controlling the magnitude of the gradients. Following the convolutional layer is a layer of batch normalization and an Exponential Linear Unit (ELU) nonlinear activation layer with *α* value of 1, which is followed by a max pooling layer having a filter and stride size of 2 in all dimensions to reduce number of feature maps size for computational efficiency. After repeating block A for five times, another block named block B is given a single time. This block contains three FC layers, one dropout layer having a probability of 10%, softmax, and a classification layer. Number of neurons in the FC layers is 100, 50, and 3 to perform multiclass (3-classes) classification task. Each of the FC layers has a weight and bias L2 factor of 0.00005 to assist in mitigating the impact of overfitting by controlling the magnitude of the gradients.

In the case of tasks involving MRI modality, the input layer takes a volume with a size of 121 × 145 × 41 while for the tasks involving PET modality, the input layer takes a volume with a size of 79 × 95 × 69. Neurons in the last FC layer are 2 for the binary classification tasks and 3 for the multiclass classification tasks.

## 4. Experimental Results

An approach of 5-fold cross-validation is employed for the hyperparameters selection. For the balanced multiclass, imbalanced multiclass, and imbalanced binary classification tasks, we considered Relative Classifier Information (RCI), Confusion Entropy (CEN), Index of Balanced Accuracy (IBA), Geometric Mean (GM), and Matthews' Correlation Coefficient (MCC) as metrics of performance. Sensitivity (SEN), Specificity (SPEC), F-measure, Precision, and Balanced Accuracy are employed as performance metrics for the balanced binary classification task.

We chose a piecewise learning rate scheduler that reduces the initial learning rate of 0.001 after every 6 epochs for experiments on all classification tasks that involve PET neuroimaging modality, as well as binary classification between AD and NC classes using MRI neuroimaging modality. Furthermore, we train the architectures for 30 epochs with a mini-batch size of 2. We employ Adam [61] as an optimizer while categorical cross entropy is used as a loss function.

For experiments on the multiclass classification tasks that involve MRI neuroimaging modality, after every 5 epochs the initial learning rate is reduced. The 3D-CNN architectures are trained for 25 epochs. For all of the experiments, we considered a mini-batch size of two. Adam is used as an optimizer, whereas the categorical cross entropy is used as a loss function. The results of the experiments are now presented in Tables 3–6.

## 5. Experiments, Results, Analysis, and Discussion

In this section, a detailed discussion about the experimental results presented in Tables 3–6 and Figures 2–9 is provided. In Table 3, the best classification model considering only the RCI performance metric is the 3D-CNN architecture using PET modality having random weak Gaussian blurred augmentation with a value of 0.2167 whereas the worst performing model is the 3D-CNN architecture using MRI modality with random width/height shift augmentation with a value of 0.052. Similarly, in terms of average CEN values, the best classification model is the 3D-CNN trained using PET modality with random zoomed in/out augmentation with a value of 0.6157 while the worst performing model is the one that employs the 3D-CNN architecture trained using MRI modality with random zoomed in/out augmentation technique with a value of 0.7069. Also, in terms of average IBA values, the best performing model is the 3D-CNN architecture trained with random zoomed in/out augmentation and PET modality with a value of 0.4165 whereas the worst performing model is the one trained using MRI modality with random width/height shift augmentation technique with a value of 0.2077. Likewise, in terms of average GM value, the best classification model is 3D-CNN architecture trained using random zoomed in/out augmentation and PET modality with a value of 0.6749 whereas the worst performing architecture is the 3D-CNN model trained using MRI modality and random width/height shift augmentation with a value of 0.5382. Finally, in terms of average MCC values, the best performing model is the 3D-CNN architecture trained using random zoomed in/out augmentation and PET modality with a value of 0.3953 while the worst performing model is the 3D-CNN architecture trained using random width/height shift augmentation and MRI neuroimaging modality.

In Table 3, a number of interesting trends are observed. We can see that 3D-CNN architectures that employed PET modality performed better than those that employed MRI modality. Overall, the best performing model is the 3D-CNN architecture trained using PET modality and random zoomed (in/out) augmentation whereas the worst performing model is the 3D-CNN architecture trained using random width/height shift augmentation and MRI neuroimaging modality. It can also be observed that combining augmentations may not result in obtaining better presentations as compared to employing single augmentation schemes.

As given in Table 4, in terms of SEN metric, the best performing model is the 3D-CNN architecture trained using PET data with random width/height shift augmentation whereas the worst performing model is the 3D-CNN architecture trained using PET data with combined random width/height shift, random zoomed (in/out), and random weak Gaussian blurred augmentations. In fact, in terms of SEN, SPEC, F-measure, Precision and Balanced Accuracy, the worst performing model is the 3D-CNN architecture trained using PET data with combined random width/height shift, random zoomed in/out, and random weak Gaussian blurred augmentation techniques. An interesting observation is the exact same performances of 3D-CNN architecture trained using PET data with random zoomed (in/out) augmentation and 3D-CNN trained using PET data with random weak Gaussian blurred augmentation, and overall, these two methods are the best when considering all the performance metrics. As can be seen, combining augmentation methods results in deteriorating performances. It can be also seen that the best model in terms of SEN and F-measure metrics is the 3D-CNN trained using PET data with random width/height shift augmentation method.

In Table 5, for binary classification between AD and NC classes using PET modality, with respect to all performance metrics, we can see that the worst performing model is the 3D-CNN architecture trained using combined random width/height shift, random zoomed in/out, and random weak Gaussian blurred augmentation methods while the best performing model, considering all the performance metrics, is the 3D-CNN architecture trained using random weak Gaussian blurred augmentation method. However, in terms of SEN metric, the best performing model is the 3D-CNN architecture trained using random width/height shift augmentation using PET modality.

Similarly, in Table 5, for binary classification between AD and NC classes using MRI modality, an interesting trend can be seen, in which RCI, average CEN, IBA, GM, and MCC metrics agree that the best classification model is the 3D-CNN architecture trained using random zoomed (in/out) augmentation method while the worst classification model is the 3D-CNN architecture trained using random weak Gaussian blurred augmentation method.

In Table 6, it can be observed that the best classification model, in terms of SEN metric, is the 3D-CNN architecture trained with random width/height shift augmentation method while the worst classification model in terms of SEN metric is the 3D-CNN architecture trained with random zoomed (in/out) augmentation method. As a matter of fact, the 3D-CNN architecture trained with random zoomed in/out augmentation method performed the worst in terms of SEN, SPEC, F-measure, accuracy, and balanced accuracy performance metrics. The best performing model is the 3D-CNN architecture trained with random weak Gaussian blurred augmentation when considering SPEC metric alone. In terms of F-measure, precision, and balanced accuracy, the 3D-CNN architecture trained with random width/height shift augmentation performed the best. We can see that combining augmentations results in suboptimal performances on this task. Overall, we found the performance of 3D-CNN architecture trained with random width/height shift augmentation method to be the best.

We have observed mixed performances in terms of different binary and the multiclass classification tasks and found random zoomed in/out augmentation to be the best performing augmentation method. We further note that architecture engineering has less impact on the final classification performance in comparison to the data manipulation schemes. Deeper architectures may not provide performance advantages in comparison with their shallower counterparts. We also found that class imbalance problem is not mitigated by data augmentation methods as for the multiclass classification task involving MRI neuroimaging modality, the final classification performance is clearly biased towards MCI class instances.

Clinical manifestations of AD are important from different perspectives. Changes associated with AD are limited to certain brain regions such as hippocampus and entorhinal cortex in the very early phases. However, as time passes, more and more brain regions are affected during this progression process. Age is perhaps the most important contributory factor as changes associated with this factor are more pronounced in subjects with higher levels of cognitive decline, followed by MCI and NC subjects. Cognitive reserve is important in considering changes associated with AD as more and more subjects have limited cognitive conscience as time passes and this affects the manifestations connected with AD [19, 62–67].

From the results, it is clear that NC-MCI binary classification is the most difficult task among the three binary classification tasks which could be due to the limited changes occurring in the brain at this stage and one of the limitations of whole brain slices is that they may fail to capture local brain changes that are associated with AD. We also found multiclass classification task to be the most difficult one among all tasks as addition of new classes usually leads to deteriorating performances if the number of samples is not appropriately handled. Methods that can capture changes at a local level are more likely to perform better on NC-MCI binary and AD-NC-MCI multiclass classification tasks.

We noted that class imbalance has a limited impact on the performances of the architectures that used MRI neuroimaging modality for AD/NC binary classification task due to almost equal number of samples in the training and validation splits. Furthermore, we noted that data augmentation cannot alleviate the class imbalance issue.

There are a number of limitations of this study such as lack of utilization of multimodal and neuropsychological information, for instance, age and other factors, which could be incorporated through FC layers inside a DL architecture and have shown to improve diagnostic performances. Furthermore, testing on an independent test set such as that based on single center studies like Open Access Series of Imaging Studies (OASIS) while training on multicentre datasets like ADNI could further boost the diagnostic performances. Tweaking the hyperparameters in an optimal way will likely improve the performance even further [68–70].

A comparison of the proposed methods with the state of the art in the literature is presented in Table 7. It can be observed that multiclass classification is the hardest task, followed by NC-MCI binary classification task, followed by AD-MCI binary classification task, and, finally, AD-NC is the easiest task.

## 6. Conclusions

In this work, we have trained different DL models in the 3D domain to study binary and multiclass classification of AD using PET and MRI neuroimaging modalities. Furthermore, we have studied the impact of random zoomed (in/out), random weak Gaussian blurred, and random width/height shift augmentation methods for different binary and multiclass classification tasks. We have found the performance of random zoomed (in/out) augmentation to be the best across all tasks. We have further noted that combining various augmentation methods results in suboptimal performances. We have also observed that architecture engineering has less of an impact on the final classification performance in comparison to data manipulation schemes such as augmentation methods. In the future, we are planning to extend this study by deploying other architectural choices such as graph convolutional networks as well as other data augmentation approaches such as elastic and plastic deformations, color jittering, and cutout augmentation.

## Figures and Tables

**Figure 1:** Architecture for processing PET and MRI scans for binary and multiclass classification tasks.

**Figure 2:** Visual representation of the results for the multiclass classification task.

**Figure 3:** Visual representation of the rankings for the multiclass classification task.

**Figure 4:** Visual representation of the results for AD-MCI binary classification task.

**Figure 5:** Visual representation of the rankings for AD-MCI binary classification task.

**Figure 6:** Visual representation of the results for AD-NC binary classification task.

**Figure 7:** Visual representation of the rankings for AD-NC binary classification task employing (a) MRI data and (b) PET data.

**Figure 8:** Visual representation of the results for MCI-NC binary classification task.

**Figure 9:** Visual representation of the rankings for MCI-NC binary classification task.

**Table 1:** PET scans of the subjects displayed in mean (min-max) format.

Research group	NC	MCI	AD
Subjects number	102	97	94
Age	76.01 (62.2–86.6)	74.54 (55.3–87.2)	75.82 (55.3–88)
Weight	75.7 (49–130.3)	77.13 (45.1–120.2)	74.12 (42.6–127.5)
FAQ total score	0.186 (0–6)	3.16 (0–15)	13.67 (0–27)
NPI-Q total score	0.402 (0–5)	1.97 (0–17)	4.074 (0–15)

FAQ : Functional Activities Questionnaire; NPI-Q : Neuropsychiatric Inventory Questionnaire.

**Table 2:** MRI scans of the subjects displayed in mean (min-max) format.

Research group	NC	MCI	AD
Number of subjects	228	396	187
Age	75.97 (60.02–89.74)	74.89 (54.63–89.38)	75.4 (55.18–90.99)
Weight	75.91 (45.81–137.44)	75.87 (43.54–121.11)	72.03 (37.65–127.46)
MMSCORE	29.11 (25–30)	27.02 (24–30)	23.26 (18–27)
CDGLOBAL score	0 (0–0)	0.5 (0–0.5)	0.75 (0.5–1)

MMSCORE : Mini-Mental Status Examination Score;CDGLOBAL : Global Clinical Dementia Rating Score.

**Table 3:** Results of multiclass classification task between AD, NC, and MCI classes.

Architecture	Performance Metrics
3D-CNN trained using PET data with random width/height shift augmentation	RCI = 0.1894, CEN = {'AD': 0.5452, 'MCI': 0.8397, 'NC': 0.5454}, Average CEN = 0.6434, IBA = {'AD': 0.4804, 'MCI': 0.1590, 'NC': 0.4505}, Average IBA = 0.3633, GM = {'AD': 0.7445, 'MCI': 0.5039, 'NC': 0.7277}, Average GM = 0.6587, MCC = {'AD': 0.4860, 'MCI': 0.077, 'NC': 0.4611} Average MCC = 0.3413
3D-CNN trained using PET data with random zoomed (in/out) augmentation	RCI = 0.2054, CEN = {'AD': 0.5088, 'MCI': 0.8038, 'NC': 0.5346}, Average CEN = 0.6157, IBA = {'AD': 0.5660, 'MCI': 0.1091, 'NC': 0.5745}, Average IBA = 0.4165, GM = {'AD': 0.7928, 'MCI': 0.4914, 'NC': 0.7406}, Average GM = 0.6749, MCC = {'AD': 0.5784, 'MCI': 0.1462, 'NC': 0.4614} Average MCC = 0.3953
3D-CNN trained using PET data with random weak Gaussian blurred augmentation	RCI = 0.2167, CEN = {'AD': 0.5051, 'MCI': 0.84, 'NC': 0.5119}, Average CEN = 0.619, IBA = {'AD': 0.4540, 'MCI': 0.1744, 'NC': 0.4270}, Average IBA = 0.3518, GM = {'AD': 0.7439, 'MCI': 0.5018, 'NC': 0.7214}, Average GM = 0.6557, MCC = {'AD': 0.4988, 'MCI': 0.0494, 'NC': 0.4561} Average MCC = 0.3347
3D-CNN trained using PET data with combined random width/height shift, random zoomed (in/out), and random weak Gaussian blurred augmentations	RCI = 0.1741, CEN = {'AD': 0.5747, 'MCI': 0.8179, 'NC': 0.5559}, Average CEN = 0.6495, IBA = {'AD': 0.4280, 'MCI': 0.1812, 'NC': 0.4851}, Average IBA = 0.3647, GM = {'AD': 0.7318, 'MCI': 0.5294, 'NC': 0.7317}, Average GM = 0.6643, MCC = {'AD': 0.4802, 'MCI': 0.1188, 'NC': 0.4572} Average MCC = 0.3520
3D-CNN trained using MRI data with random width/height shift augmentation	RCI = 0.052, CEN = {'AD': 0.6948, 'MCI': 0.6945, 'NC': 0.6663}, Average CEN = 0.6852, IBA = {'AD': 0.1308, 'MCI': 0.312, 'NC': 0.1804}, Average IBA = 0.2077, GM = {'AD': 0.542, 'MCI': 0.5148, 'NC': 0.5578}, Average GM = 0.5382, MCC = {'AD': 0.2477, 'MCI': 0.0455, 'NC': 0.20006}, Average MCC = 0.16442
3D-CNN trained using MRI data with random zoomed (in/out) augmentation	RCI = 0.0603, CEN = {'AD': 0.7242, 'MCI': 0.7277, 'NC': 0.6689}, Average CEN = 0.7069, IBA = {'AD': 0.1708, 'MCI': 0.2809, 'NC': 0.2768}, Average IBA = 0.2428, GM = {'AD': 0.5684, 'MCI': 0.5325, 'NC': 0.6185}, Average GM = 0.5731, MCC = {'AD': 0.2418, 'MCI': 0.0651, 'NC': 0.2615}, Average MCC = 0.1894
3D-CNN trained using MRI data with random weak Gaussian blurred augmentation	RCI = 0.0687, CEN = {'AD': 0.6473, 'MCI': 0.6869, 'NC': 0.6213}, Average CEN = 0.6518, IBA = {'AD': 0.1146, 'MCI': 0.3181, 'NC': 0.2112}, Average IBA = 0.2146, GM = {'AD': 0.5280, 'MCI': 0.5139, 'NC': 0.5906}, Average GM = 0.5441, MCC = {'AD': 0.2473, 'MCI': 0.0489, 'NC': 0.2550}, Average MCC = 0.1837

**Table 4:** Results of binary classification task between AD and MCI classes.

Architecture	Performance Metrics
3D-CNN trained using PET data with random width/height shift augmentation	SEN = 0.6702, SPEC = 0.6804, F-measure = 0.6702, Precision = 0.6702, Balanced Accuracy = 0.6753
3D-CNN trained using PET data with random zoomed in/out augmentation	SEN = 0.6277, SPEC = 0.7423, F-measure = 0.6629, Precision = 0.7024, Balanced Accuracy = 0.6850
3D-CNN trained using PET data with random weak Gaussian blurred augmentation	SEN = 0.6277, SPEC = 0.7423, F-measure = 0.6629, Precision = 0.7024, Balanced Accuracy = 0.6850
3D-CNN trained using PET data with combined random width/height shift, random zoomed (in/out), and random weak Gaussian blurred augmentations	SEN = 0.6170, SPEC = 0.7113, F-measure = 0.6444, Precision = 0.6744, Balanced Accuracy = 0.6642

**Table 5:** Results of binary classification task between AD and NC classes.

Architecture	Performance Metrics
3D-CNN trained using PET data with random width/height shift augmentation	SEN = 0.8404, SPEC = 0.8725, F-measure = 0.8495, Precision = 0.8587, Balanced Accuracy = 0.8565
3D-CNN trained using PET data with random zoomed (in/out) augmentation	SEN = 0.8298, SPEC = 0.8627, F-measure = 0.8387, Precision = 0.8478, Balanced Accuracy = 0.8463
3D-CNN trained using PET data with random weak Gaussian blurred augmentation	SEN = 0.8404, SPEC = 0.8922, F-measure = 0.8587, Precision = 0.8778, Balanced Accuracy = 0.8663
3D-CNN trained using PET data with combined random width/height shift, random zoomed (in/out), and random weak Gaussian blurred augmentations	SEN = 0.8191, SPEC = 0.8431, F-measure = 0.8235, Precision = 0.8280, Balanced Accuracy = 0.8311
3D-CNN trained using MRI data with random width/height shift augmentation	RCI = 0.2210, CEN = {'AD': 0.7421, 'NC': 0.6923}, Average CEN = 0.7172, IBA = {'AD': 0.6054, 'NC': 0.5794}, Average IBA = 0.5924, GM = {'AD': 0.7697, 'NC': 0.7697}, Average GM = 0.7697, MCC = {'AD': 0.5371, 'NC': 0.5371}, Average MCC = 0.5371
3D-CNN trained using MRI data with random zoomed in/out augmentation	RCI = 0.25, CEN = {'AD': 0.7319, 'NC': 0.6455}, Average CEN = 0.6887, IBA = {'AD': 0.5701, 'NC': 0.6579}, Average IBA = 0.614, GM = {'AD': 0.7836, 'NC': 0.7836}, Average GM = 0.7836, MCC = {'AD': 0.5707, 'NC': 0.5707}, Average MCC = 0.5707
3D-CNN trained using MRI data with random weak Gaussian blurred augmentation	RCI = 0.2145, CEN = {'AD': 0.7687, 'NC': 0.6739}, Average CEN = 0.7213, IBA = {'AD': 0.5263, 'NC': 0.6365}, Average IBA = 0.5814, GM = {'AD': 0.7625, 'NC': 0.7625}, Average GM = 0.7625, MCC = {'AD': 0.5311, 'NC': 0.5311}, Average MCC = 0.5311

**Table 6:** Results of binary classification task between NC and MCI classes.

Architecture	Performance Metrics
3D-CNN trained with PET data using random width/height shift augmentation	SEN = 0.5876, SPEC = 0.6569, F-measure = 0.6032, Precision = 0.6196, Balanced Accuracy = 0.6222
3D-CNN trained with PET data using random zoomed (in/out) augmentation	SEN = 0.4948, SPEC = 0.6569, F-measure = 0.5333, Precision = 0.5783, Balanced Accuracy = 0.5759
3D-CNN trained with PET data using random weak Gaussian blurred augmentation	SEN = 0.5464, SPEC = 0.6765, F-measure = 0.5792, Precision = 0.6163, Balanced Accuracy = 0.6114
3D-CNN trained using PET data with combined random width/height shift, random zoomed (in/out), and random weak Gaussian blurred augmentations	SEN = 0.5052, SPEC = 0.6765, F-measure = 0.5475, Precision = 0.5976, Balanced Accuracy = 0.5908

**Table 7:** Performance comparison between the proposed and the state-of-the-art methods.

Author	Data	Method	Accuracy (%)	Classification task
Oh et al. [71]	MRI	Inception autoencoder based CNN architecture	84.5	AD/NC binary classification
Yagis et al. [72]	MRI	3D-CNN architectures	73.4	AD/NC binary classification
Ieracitano et al. [73]	MRI	Electroencephalographic signals	85.78	AD/NC binary classification
Prajapati et al. [74]	MRI	DL model employing FC layers	85.19	AD/NC binary classification
Tomassini et al. [75]	MRI	3D convolutional long short-term memory based network	86	AD/NC binary classification
Rejusha et al. [76]	MRI	Deep convolutional GAN	83	AD/NC binary classification
Yagis et al. [77]	MRI	2D CNN autoencoder architecture	74.66	AD/NC binary classification
Sarasua et al. [78]	Functional MRI	Template based DL architecture	77.3	AD/NC binary classification
Fedorov et al. [79]	MRI	Multimodal architectures	84.1	AD/NC binary classification
**Our approach (random weak Gaussian blurred augmentation)**	**PET**	**3D-CNN whole brain**	**86.63**	**AD/NC binary classification**
Aderghal et al. [80]	MRI	2D-CNN hippocampal region	66.5	AD/MCI binary classification
Karim Aderghal et al. [81]	MRI	2D-CNN coronal, sagittal, and axial projections	63.28	AD/MCI binary classification
**Our approach (random zoomed in/out augmentation)**	**PET**	**3D-CNN whole brain**	**68.5**	**AD/MCI binary classification**
Kam et al. [82]	Resting-state functional MRI	CNN framework	73.85	NC/MCI binary classification
Ben Ahmed et al. [83]	MRI	Circular harmonic functions	69.45	NC/MCI binary classification
**Our approach (random width/height augmentation)**	**PET**	**3D-CNN whole brain**	**62.22**	**NC/MCI binary classification**
Khagi et al. [84]	PET, MRI	DL architecture employing 3D-CNN layers	50.21	AD/NC/MCI multiclass classification
Puspaningrum et al. [85]	MRI	Deep CNN architecture having three convolutional layers	55.27	AD/NC/MCI multiclass classification
**Our approach (random zoomed in/out augmentation)**	**PET**	**3D-CNN whole brain**	**59.73**	**AD/NC/MCI multiclass classification**

PET stands for Positron Emission Tomography, CNN stands for Convolutional Neural Network, AD stands for Alzheimer's disease, NC stands for Normal Control or Cognitively Normal, and MCI stands for Mild Cognitive Impairment.

## Data Availability

The data are publicly available at https://adni.loni.usc.edu.
